# Global Stability of an HIV-1 Infection Model with General Incidence Rate and Distributed Delays

**DOI:** 10.1155/2014/260379

**Published:** 2014-10-29

**Authors:** Abdoul Samba Ndongo, Hamad Talibi Alaoui

**Affiliations:** Department of Mathematics and Informatics, Faculty of Sciences, Chouaib Doukkali University, BP 20, 24000 El Jadida, Morocco

## Abstract

In this work an HIV-1 infection model with nonlinear incidence rate and distributed intracellular delays and with humoral immunity is investigated. The disease transmission function is assumed to be governed by general incidence rate *f*(*T*, *V*)*V*. The intracellular delays describe the time between viral entry into a target cell and the production of new virus particles and the time between infection of a cell and the emission of viral particle. Lyapunov functionals are constructed and LaSalle invariant principle for delay differential equation is used to establish the global asymptotic stability of the infection-free equilibrium, infected equilibrium without *B* cells response, and infected equilibrium with *B* cells response. The results obtained show that the global dynamics of the system depend on both the properties of the general incidence function and the value of certain threshold parameters *R*_0_ and *R*_1_ which depends on the delays.

## 1. Introduction

Immunity can be broadly categorized into adaptive immunity and innate immunity. Adaptive immunity is mediated by clonally distributed *T* and *B* lymphocytes, namely, humoral and cellular immunity, and is characterized by specificity and memory. The humoral immunity plays an important role in antiviral defence by attacking virus. A basic mathematical model describing HIV-1 infection dynamics model with humoral immunity was introduced by Murase et al. [1] as

(1) $$\begin{array}{c} \frac{dT\left(t\right)}{dt}=\Lambda -dT\left(t\right)-\beta T\left(t\right)V\left(t\right),\\ \frac{dI\left(t\right)}{dt}=\beta T\left(t\right)V\left(t\right)-\delta I\left(t\right),\\ \frac{dV\left(t\right)}{dt}=N\delta I\left(t\right)-cV\left(t\right)-qB\left(t\right)V\left(t\right),\\ \frac{dB\left(t\right)}{dt}=gB\left(t\right)V\left(t\right)-\mu B\left(t\right), \end{array}$$

where *T*(*t*), *I*(*t*), *V*(*t*), and *B*(*t*) represent the densities of uninfected cells, infected cells, virus, and *B* cells at time *t*, respectively. Λ and *d* are the birth and death rate constants of uninfected cells. *β* is the infection rate, *N* is the average number of virus particles produced over the lifetime of a single infected cells, and *δ* is the death rate of infected cells; *c* is the death rate constant of the virus, *g* and *μ* are the recruited rate and death rate constants of *B* cells, and *q* is the *B* cells neutralization rate. Mathematical models for virus dynamics with antibody immune response has drawn much attention of researchers (see, e.g., [1–13] and the reference therein). Recently many studies have been done to improve the model (1) by introducing delays and changing the incidence rate according to different practical background. These studies used different delayed models with different forms of incidence rate; see, for example, [6, 9–11] for discrete delays and [5, 13] for distributed delays.

In the present paper, motivated by the works of [1, 5, 13], we propose the following model with a general incidence rate and distributed delays and humoral immunity:

(2) dTtdt=Λ−dTt−fTt,VtVt,dItdt=∫0h1P1τe−m1τfTt−τ,Vt−τ ×Vt−τdτ−δIt,dVtdt=Nδ∫0h2P2τe−m2τIt−τdτ −cV(t)−qB(t)V(t),dBtdt=gBtVt−μBt,

where the parameters in system (2) have the same meanings as in system (1). *f*(*T*, *V*)*V* is the general incidence rate. It is assumed in (2) that the uninfected cells that are contacted by the virus particles at time *t* − *τ* become infected cells at time *t*, where *τ* is distributed according to *P*_1_(*τ*) over the interval [0, *h*_1_], where *h*_1_ is the limit superior of this delay. The constant *m*_1_  (*m*_1_ > 0) is assumed to be the death rate for infected cells during time period [*t* − *τ*, *t*] but not yet virus-producing cells and the term *e* ^−*m*_1_*τ*^ denotes the surviving rate of infected cells during the delay period. On the other hand, it is assumed in (2) that a cell infected at time *t* − *τ* starts to yield new infectious virus at time *t*, where *τ* is distributed according to a probability distribution *P*_2_(*τ*) over the interval [0, *h*_2_] and *h*_2_ is limit superior of this delay. The factor *e* ^−*m*_2_*τ*^ accounts for the probability of surviving infected cells during the time period of delay, where *m*_2_ is constant. In (2), the probability distribution functions *P*_*i*_(*τ*), *i* = 1,2, are assumed to satisfy *P*_*i*_(*τ*) > 0, *i* = 1,2 and

(3) $$\begin{array}{c} \overset{h_{i}}{\underset{0}{\int }}P_{i}\left(\tau \right)d\tau =1,\;\overset{h_{i}}{\underset{0}{\int }}\tau P_{i}\left(\tau \right)d\tau <\infty ,\;i=1,2. \end{array}$$

The function *f* is assumed to be continuously differentiable in the interior of *IR*_+_^2^ and satisfies the following hypotheses:

(*H*_1_) *f*(0, *V*) = 0, for all *V* ≥ 0,
(*H*_2_) ∂*f*(*T*, *V*)/∂*T* > 0, for all *T* > 0 and *V* ≥ 0,
(*H*_3_) ∂*f*(*T*, *V*)/∂*V* ≤ 0, for all *T* > 0 and *V* ≥ 0.
(*H*_4_) ∂(*f*(*T*, *V*)*V*)/∂*V* ≥ 0, for all *T*, *V* > 0.

The biological meaning of hypothesis (*H*_1_) to (*H*_4_) is given in [10].

Note the following.

The incidence rate *f*(*T*, *V*)*V* given in (2) generalizes many common forms such as [5, 9, 13] (see Section 6).

The distributed delay is more general than the discrete one and it is more adapted to biological phenomena.

*h*_1_ or *h*_2_ can be infinity.

The present paper is organized as follows. In Section 2, we establish the nonnegativity and boundedness of solutions and we derived the basic reproduction ratios for viral infection and humoral immune response *R*_0_ and *R*_1_, respectively. In Section 3, the existence of a possible three positive equilibria, an infection-free equilibrium *E*_0_^*^, an infected equilibrium without *B* cells response *E*_1_^*^, and an infected equilibrium with *B* cells response *E*_2_^*^, is established. In Sections 4 and 5, we show that the global asymptotic stability of these equilibria depend only on the basic reproduction numbers under some hypotheses on the incidence function. In Section 6, some examples are given. A brief discussion is given in the last section to conclude this paper.

## 2. Preliminary Results

The initial conditions of (2) are given as

(4) Tθ=ϕ1θ,  Iθ=ϕ2θ,    Vθ=ϕ3θ,Bθ=ϕ4θ,ϕiθ≥0, i=1,2,3,4,θ∈−h,0,    h=max⁡h1,h2,

where *ϕ* = (*ϕ*_1_, *ϕ*_2_, *ϕ*_3_, *ϕ*_4_) ∈ *C* ^+^, here *C* ^+^ = *C*(−*h*, 0], *ℜ*_+_^4^), with *C*(−*h*, 0], *ℜ* ^4^); denotes the Banach space of continuous functions mapping the interval −*h*, 0] into *ℜ* ^4^.

**Theorem 1 .**

Under the initial conditions (4), all solutions (*T*(*t*), *I*(*t*), *V*(*t*), *B*(*t*)) of system (2) are nonnegative on [0, +*∞* and bounded.

**Proof**

Let us put system (2) in a vector form by setting *Z* = (*T*, *I*, *V*, *B*)^*T*^ and

(5) GZ=G1ZG2ZG3ZG3Z=Λ−dTt−fTt,VtVt∫0h1P1τe−m1τfTt−τ,Vt−τVt−τdτ−δItNδ∫0h2P2τe−m2τIt−τdτ−cVt−qBtVtgBtVt−μBt,

where *G* : *C*_+_ → *IR* ^4^ and *C*_+_ = {*ϕ* = (*ϕ*_1_, *ϕ*_2_, *ϕ*_3_, *ϕ*_4_) : *ϕ* ∈ *C*([−*h*, 0], *IR*_+_^4^)}. It is easy to check that *G*_*i*_(*Z*)∣_*Z*_*i*_=0_ ≥ 0, *i* = 1,2, 3,4. Due to [14, Lemma  2], any solution of (2) with *Z*(*θ*) ∈ *C*_+_, say *Z*(*t*) = *Z*(*t*, *Z*(*θ*)), is such that *Z*(*t*) ∈ *IR*_+_^4^ for all *t* ≥ 0. Next we show that the solutions are also bounded. It follows from the first equation of (2) that *dT*/*dt* ≤ Λ − *dT*(*t*). This implies lim⁡ sup⁡_*t*→*∞*_ *T*(*t*) ≤ Λ/*d*, so *T*(*t*) is bounded.

Let

(6) $$\begin{array}{c} F\left(t\right)=\overset{h_{1}}{\underset{0}{\int }}P_{1}\left(\tau \right)e^{-m_{1}\tau }T\left(t-\tau \right)d\tau +I\left(t\right). \end{array}$$

Then

(7) dFtdt=Λ∫0h1P1τe−m1τdτ−d∫0h1P1τe−m1τTt−τdτ −δIt≤Λ−γFt,

where *γ* = min⁡{*d*, *δ*} and thus lim⁡ sup⁡_*t*→*∞*_ *F*(*t*) ≤ Λ/*γ*. This implies that *F*(*t*) is bounded and so is *I*(*t*). Thus, there exists a *χ* > 0 such that *I*(*t*) ≤ *χ*. It follows from the third equations in (2) that

(8) $$\begin{array}{c} \frac{dV\left(t\right)}{dt}\leq N\delta \chi -cV\left(t\right), \end{array}$$

and consequently *V*(*t*) is bounded. On the other hand, let

(9) $$\begin{array}{c} H\left(t\right)=V\left(t\right)+\frac{q}{g}B\left(t\right). \end{array}$$

Then,

(10) $$\begin{array}{c} \frac{dH\left(t\right)}{dt}=N\delta \overset{h_{2}}{\underset{0}{\int }}P_{2}\left(\tau \right)e^{-m_{2}\tau }I\left(t-\tau \right)d\tau -cV\left(t\right)-\frac{q\mu }{g}B\left(t\right). \end{array}$$

We have *dH*(*t*)/*dt* ≤ *Nδχ* − *ξH*(*t*), where *ξ* = min⁡{*c*, *μ*}; this implies that *H*(*t*) is bounded so also for *B*(*t*). Finally, all the solutions of system (2) are bounded. This completes the proof.

To simplify the notations we note that

(11) $$\begin{array}{c} k_{1}=\overset{h_{1}}{\underset{0}{\int }}P_{1}\left(\tau \right)e^{-m_{1}\tau }d\tau ,\;\;k_{2}=\overset{h_{2}}{\underset{0}{\int }}P_{2}\left(\tau \right)e^{-m_{2}\tau }d\tau . \end{array}$$

Global behaviour of system (2) may depend on the basic reproduction numbers *R*_0_ and *R*_1_ given by

(12) $$\begin{array}{c} R_{0}=\frac{Nk_{1}k_{2}f\left(T_{0}^{*},0\right)}{c}, \end{array}$$

where *T*_0_^*^ = Λ/*d* and

(13) $$\begin{array}{c} R_{1}=\frac{Nk_{1}k_{2}f\left(M,\mu /g\right)}{c}, \end{array}$$

with, *M* = *T*_0_^*^ − (*μc*/*dNgk*_1_ *k*_2_). Here, *R*_0_ and *R*_1_ are the basic reproduction ratios for viral infection and humoral immune response of system (2), respectively. Based on the hypotheses (*H*_2_) and (*H*_3_) it is clear that *R*_1_ < *R*_0_.

## 3. The Existence of Positive Equilibria

In this section we prove the existence of positive equilibrium. The system (2) always has an infection-free equilibrium *E*_0_^*^ = (*T*_0_^*^, 0,0, 0). For other possible equilibriums, we have the following theorem.

**Theorem 2 .**

Suppose that the conditions (H_1_)–(H_3_) are satisfied.

(1) If *R*_0_ > 1, then system (2) has an infected equilibrium without *B* cells response of the form *E*_1_^*^ = (*T*_1_^*^, *I*_1_^*^, *V*_1_^*^, 0) with *T*_1_^*^ ∈ (0, *T*_0_^*^).
(2) If *R*_1_ > 1, then system (2) has an infected equilibrium with *B* cells response of the form *E*_2_^*^ = (*T*_2_^*^, *I*_2_^*^, *V*_2_^*^, *B*_2_^*^) with *T*_2_^*^ ∈ (0, *M*).

**Proof**

The steady states of system (2) satisfy the following equations:

(14) $$\begin{array}{c} \Lambda -dT-f\left(T,V\right)V=0,\\ k_{1}f\left(T,V\right)V-\delta I=0,\\ N\delta k_{2}I-cV-qBV=0,\\ gBV-\mu B=0. \end{array}$$

From the last equation of (14), we have

(15) $$\begin{array}{c} \left(gV-\mu \right)B=0. \end{array}$$

Equations (15) has two possible solutions, *B* = 0 or *gV* − *μ* = 0.

If *B* = 0, (14)_3_ yields *I* = (*c*/*Nδk*_2_)*V*.

By substituting this into (14)_2_, we obtain that

(16) $$\begin{array}{c} \left(k_{1}f\left(T,V\right)-\frac{c}{Nk_{2}}\right)V=0, \end{array}$$

which gives *V* = 0 or *k*_1_ *f*(*T*, *V*) − (*c*/*Nk*_2_) = 0.

If *V* = 0, we obtain the infection-free equilibrium *E*_0_^*^(Λ/*d*, 0,0, 0).

If *V* ≠ 0, (14)_1_ and (14)_2_ yields

(17) $$\begin{array}{c} I=\frac{k_{1}\left(\Lambda -dT\right)}{\delta }≔I\left(T\right). \end{array}$$

By substituting this into (14)_3_, we obtain

(18) $$\begin{array}{c} V=\frac{Nk_{1}k_{2}\left(\Lambda -dT\right)}{c}≔V\left(T\right). \end{array}$$

Since *I* ≥ 0 and *V* ≥ 0, this implies that *T* ≤ Λ/*d*.

Now, from (*H*_1_), (*H*_2_), and (*H*_3_), the following functional

(19) $$\begin{array}{c} K\left(T\right)=k_{1}f\left(T,V\left(T\right)\right)-\frac{c}{Nk_{2}}, \end{array}$$

satisfies

(20) $$\begin{array}{c} K\left(0\right)K\left(\frac{\Lambda }{d}\right)=-{\left(\frac{c}{Nk_{2}}\right)}^{2}\left(R_{0}-1\right)<0,\;\text{for}\;\;R_{0}>1,\\ \dot{K}\left(T\right)=k_{1}\frac{\partial f}{\partial T}-\frac{Ndk_{1}k_{2}}{c}\frac{\partial f}{\partial V}>0. \end{array}$$

Hence, we obtain the infected equilibrium without *B* cells response

(21) $$\begin{array}{c} E_{1}^{*}=\left(T_{1}^{*},I_{1}^{*},V_{1}^{*},0\right)=\left(T_{1}^{*},I\left(T_{1}^{*}\right),V\left(T_{1}^{*}\right),0\right), \end{array}$$

where *T*_1_^*^ is the unique zero in (0, *T*_0_^*^) of *K* and *I* and *V* are given by (17) and (18).

If *B* ≠ 0, from (15), we obtain

(22) $$\begin{array}{c} V=\frac{\mu }{g}≔V_{2}^{*}, \end{array}$$

and from the first and second equation of (14), we have

(23) $$\begin{array}{c} I=I\left(T\right)=\frac{k_{1}\left(\Lambda -dT\right)}{\delta }\geq 0. \end{array}$$

By substituting this into (14)_3_, we obtain

(24) $$\begin{array}{c} B=B\left(T\right)=\frac{dNgk_{1}k_{2}\left(M-T\right)}{q\mu }\geq 0, \end{array}$$

which implies that *T* ≤ *M*.

Now, from (14)_1_ the functional

(25) $$\begin{array}{c} L\left(T\right)≔\Lambda -dT-f\left(T,V_{2}^{*}\right)V_{2}^{*}=0 \end{array}$$

satisfies

(26) $$\begin{array}{c} L\left(0\right)L\left(M\right)=\Lambda \left(\frac{\mu c}{Ngk_{1}k_{2}}\right)\left(1-R_{1}\right)<0,\;\text{for}\;\;R_{1}>1\\ \dot{L}\left(T\right)=-\frac{\mu }{g}\frac{\partial f}{\partial T}-d<0. \end{array}$$

Hence, we obtain the infected equilibrium with *B* cells response *E*_2_^*^ = (*T*_2_^*^, *I*(*T*_2_^*^), *V*_2_^*^, *B*(*T*_2_^*^)), where *T*_2_^*^ is the unique zero of *L* in (0, *M*) and *I* and *B* are given by (23) and (24), respectively. This completes the proof.

**Remark 3 .**

From (19) we have *K*(*M*) = (*c*/*Nk*_2_)(*R*_1_ − 1) ≤ 0 if *R*_1_ ≤ 1. So, as *K* is increasing in the interval [*o*, Λ/*d*], we deduces that *M* ≤ *T*_1_^*^ and consequently *V*_1_^*^ − (*μ*/*g*) ≤ 0.

## 4. Global Stability of the Infection-Free Equilibrium

In this section, we study the global stability of the infection-free equilibrium *E*_0_^*^ of system (2).

**Theorem 4 .**

Suppose that the conditions (H_1_)–(H_3_) are satisfied. Then the infection-free equilibrium *E*_0_^*^ of system (2) is globally asymptotically stable if *R*_0_ ≤ 1.

**Proof**

Define a Lyapunov functional:

(27) U0t=∫T0∗T1−fT0∗,0fσ,0dσ+1k1I+1Nk1k2V +qNgk1k2B+1k1∫0h1P1τe−m1τ ×∫t−τtfTσ,VσVσdσdτ +δk1k2∫0h2P2τe−m2τ∫t−τtIσdσdτ,

where *k*_1_ and *k*_2_ are given in (11).

It is obvious that *U*_0_ is defined and continuously differentiable for all *T*, *I*, *V*, B > 0, and *U*_0_ = 0 at *E*_0_^*^. The time derivative of *U*_0_(*t*) along the solutions of system (2) is given by

(28) U˙0=1−fT0∗,0fT,0Λ−dT−fT,VV +1k1∫0h1P1τe−m1τfTτ,VτVτdτ−δk1I +1Nk1k2Nδ∫0h2P2τe−m2τIτdτ−cV−qBV +qNgk1k2gBV−μB +1k1∫0h1P1τe−m1τfT,VV−fTτ,VτVτdτ +δk1k2∫0h2P2τe−m2τI−Iτdτ,

with *T*_*τ*_ = *T*(*t* − *τ*), *T* = *T*(*t*), *I*_*τ*_ = *I*(*t* − *τ*), *I* = *I*(*t*), *V*_*τ*_ = *V*(*t* − *τ*), *V* = *V*(*t*), and *B* = *B*(*t*).

At *E*_0_^*^, using Λ = *dT*_0_^*^, we obtain

(29) U˙0=1−fT0∗,0fT,0dT0∗−dT+fT,VVfT0∗,0fT,0 −cNk1k2V−μqNgk1k2B=d1−fT0∗,0fT,0T0∗−T+cNk1k2 ×fT,VfT,0Nk1k2fT0∗,0c−1V−μqNgk1k2B.

From (*H*_2_) and (*H*_3_) we have, respectively,

(30) 1−f(T0∗,0)f(T,0)T0∗−T≤0,fT,VfT,0Nk1k2fT0∗,0c≤fT,0fT,0Nk1k2fT0∗,0c=Nk1k2fT0∗,0c=R0.

Then, *R*_0_ ≤ 1 ensures that ${\dot{U}}_{0}\leq 0$, for all *T*, *I*, *V*, *B* ≥ 0, ${\dot{U}}_{0}=0$ holds only for *T* = *T*_0_^*^, *V* = *B* = 0, and from (2)_2_ we obtain *I* = 0. It follows that {*E*_0_^*^} is the largest invariant set in $\left\{\left(T,I,V,B\right)|{\dot{U}}_{0}=0\right\}$. It follows from LaSalle invariance principle [15] that the infection-free equilibrium *E*_0_^*^ is globally asymptotically stable.

## 5. Global Stability of the Infected Equilibria 

In this section, we study the global stability of the infected equilibrium without *B* cells response *E*_1_^*^ and the infected equilibrium with *B* cells response *E*_2_^*^ of system (2) by the Lyapunov direct method.

We set

(31) $$\begin{array}{c} g\left(x\right)=x-1-\ln x,\;\text{for}\;\;x\in \left(0,\infty \right). \end{array}$$

It is clear that for any *x* > 0, *g*(*x*) ≥ 0 and *g*(*x*) has the global minimum *x* = 1, with *g*(1) = 0.

**Theorem 5 .**

Suppose that the conditions (*H*_1_)–(*H*_4_) are satisfied. Then the equilibrium *E*_1_^*^ is globally asymptotically stable if *R*_1_ ≤ 1 < *R*_0_.

**Proof**

Define a Lyapunov functional

(32) $$\begin{array}{c} U_{1}=W_{1}+W_{2}, \end{array}$$

where

(33) W1=∫T1∗T1−fT1∗,V1∗fσ,V1∗dσ+1k1I1∗gII1∗ +V1∗Nk1k2gVV1∗+qNgk1k2B,W2=1k1fT1∗,V1∗V1∗∫0h1P1τe−m1τ ×∫t−τtgfTσ,VσVσfT1∗,V1∗V1∗dσdτ +δk1k2I1∗∫0h2P2(τ)e−m2τ∫t−τtg(I(σ)I1∗)dσdτ,

where *k*_1_ and *k*_2_ are given in (11).

The function *U* : *T* → ∫_*T*_1_^*^_^T^(1 − *f*(*T*_1_^*^, *V*_1_^*^)/*f*(*σ*, *V*_1_^*^))*dσ* verifies

(34) $$\begin{array}{c} \dot{U}\left(T\right)=1-\frac{f\left(T_{1}^{*},V_{1}^{*}\right)}{f\left(T,V_{1}^{*}\right)}. \end{array}$$

From (*H*_2_), we have $\dot{U}(T)<0$ for *T* ∈ (0, *T*_1_^*^), $\dot{U}(T)>0$ for *T* ∈ (*T*_1_^*^, *∞*), and $\dot{U}\left(T_{1}^{*}\right)=0$, so *U*(*T*) ≥ 0. Consequently *U*_1_ is nonnegative defined with respect to the endemic equilibrium *E*_1_^*^, which is a global minimum.

We now prove that the time derivative of *U*_1_ is nonpositive. Calculating the time derivative of *W*_1_ along the positive solutions of (2), we obtain

(35) W˙1=1−f(T1∗,V1∗)f(T,V1∗)T˙+1k1(1−I1∗I)I˙ +1Nk1k21−V1∗VV˙+qNgk1k2B˙=1−fT1∗,V1∗fT,I1∗,V1∗(Λ−dT−f(T,V)V) +1k11−I1∗I ×∫0h1P1(τ)e−m1τf(Tτ,Vτ)Vτdτ−δI +1Nk1k21−V1∗V ×Nδ∫0h2P2τe−m2τIτdτ−cV−qBV +qNgk1k2gBV−μB.

At *E*_1_^*^, by using Λ = *dT*_1_^*^ + *f*(*T*_1_^*^, *V*_1_^*^)*V*_1_^*^ and *c* = *Nδk*_2_ *I*_1_^*^/*V*_1_^*^ and *δ*/*k*_1_ *I*_1_^*^ = *f*(*T*_1_^*^, *V*_1_^*^)*V*_1_^*^, we have

(36) W˙1=1−f(T1∗,V1∗)f(T,V1∗)dT1∗−dT +f(T1∗,V1∗)V1∗1−f(T1∗,V1∗)f(T,V1∗) −f(T,V)V+fT1∗,V1∗fT,V1∗f(T,V)V +1k1∫0h1P1τe−m1τfTτ,VτVτdτ−δk1I −1k1I1∗I∫0h1P1τe−m1τfTτ,VτVτdτ +δk1I1∗+δk1k2∫0h2P2τe−m2τIτdτ−δI1∗k1V1∗V −δk1k2V1∗V∫0h2P2(τ)e−m2τIτdτ+δk1I1∗ +qNk1k2V1∗−μgB.

Calculating the time derivative of *W*_2_, we obtain

(37) W˙2=1k1fT1∗,V1∗V1∗∫0h1P1τe−m1τ ×fT,VVfT1∗,V1∗V1∗−fTτ,VτVτfT1∗,V1∗V1∗ hhh+ln⁡fTτ,VτVτfT,VVdτ +δk1k2I1∗∫0h2P2τe−m2τII1∗−IτI1∗+ln⁡IτIdτ=fT,VV−1k1∫0h1P1τe−m1τfTτ,VτVτdτ +1k1fT1∗,V1∗V1∗∫0h1P1τe−m1τln⁡fTτ,VτVτfT,VVdτ +δk1I−δk1k2∫0h2P2τe−m2τIτdτ +δk1k2I1∗∫0h2P2τe−m2τln⁡IτIdτ.

Combining (36) and (37) and by using (*δ*/*k*_1_)*I*_1_^*^ = *f*(*T*_1_^*^, *V*_1_^*^)*V*_1_^*^, we obtain

(38) U˙1=1−f(T1∗,V1∗)f(T,V1∗)dT1∗−dT +f(T1∗,V1∗)V1∗1−f(T1∗,V1∗)f(T,V1∗) +f(T1∗,V1∗)f(T,V1∗)f(T,V)V −1k1I1∗I∫0h1P1(τ)e−m1τf(Tτ,Vτ)Vτdτ +f(T1∗,V1∗)V1∗−f(T1∗,V1∗)V −1k2fT1∗,V1∗V1∗I1∗V1∗V∫0h2P2(τ)e−m2τIτdτ +f(T1∗,V1∗)V1∗+1k1f(T1∗,V1∗)V1∗ ×∫0h1P1(τ)e−m1τln⁡f(Tτ,Vτ)Vτf(T,V)Vdτ +1k2f(T1∗,V1∗)V1∗∫0h2P2(τ)e−m2τln⁡IτIdτ +qNk1k2V1∗−μgB=1−fT1∗,V1∗fT,V1∗dT1∗−dT +fT1∗,V1∗V1∗fT,V1∗fT,V−VV1∗ ×1−fT,VfT,V1∗+fT1∗,V1∗V1∗ ×1−fT1∗,V1∗fT,V1∗+ln⁡fT1∗,V1∗fT,V1∗ +fT1∗,V1∗V1∗1−fT,V1∗fT,V+ln⁡fT,V1∗fT,V +1k1f(T1∗,V1∗)V1∗∫0h1P1(τ)e−m1τ ×1−fTτ,VτVτI1∗fT1∗,V1∗V1∗I+ln⁡fTτ,VτVτI1∗fT1∗,V1∗V1∗Idτ +1k2f(T1∗,V1∗)V1∗∫0h2P2(τ)e−m2τ ×1−IτV1∗I1∗V+ln⁡IτV1∗I1∗Vdτ+qNk1k2V1∗−μgB=d1−f(T1∗,V1∗)f(T,V1∗)T1∗−T +fT1∗,V1∗V1∗fT,V1∗fT,V−VV1∗1−fT,VfT,V1∗ −f(T1∗,V1∗)V1∗g(fT1∗,V1∗fT,V1∗)−f(T1∗,V1∗)V1∗g ×fT,V1∗fT,V−1k1f(T1∗,V1∗)V1∗ ×∫0h1P1(τ)e−m1τg(f(Tτ,Vτ)VτI1∗f(T1∗,V1∗)V1∗I)dτ −1k2f(T1∗,V1∗)V1∗∫0h2P2(τ)e−m2τgIτV1∗I1∗Vdτ +qNk1k2V1∗−μgB.

From (*H*_2_), we have

(39) $$\begin{array}{c} \left(1-\frac{f\left(T_{1}^{*},V_{1}^{*}\right)}{f\left(T,V_{1}^{*}\right)}\right)\left(T_{1}^{*}-T\right)\leq 0, \end{array}$$

and from (*H*_3_) and (*H*_4_) we have

(40) $$\begin{array}{c} \left(\frac{f\left(T,V_{1}^{*}\right)}{f\left(T,V\right)}-\frac{V}{V_{1}^{*}}\right)\left(1-\frac{f\left(T,V\right)}{f\left(T,V_{1}^{*}\right)}\right)\leq 0, \end{array}$$

and as *g* is positive, we have

(41) $$\begin{array}{c} {\dot{U}}_{1}\leq \frac{q}{Nk_{1}k_{2}}\left(V_{1}^{*}-\frac{\mu }{g}\right)B. \end{array}$$

From Remark 3 we have ${\dot{U}}_{1}\left(t\right)\leq 0$ for all *T*, *I*, *V*, *B* ≥ 0. It is easy to verify that from (38), the largest invariant set in $\left\{\left(T,I,V,B\right)\setminus {\dot{U}}_{1}\left(t\right)=0\right\}$ is the singleton {*E*_1_^*^}. Using LaSalle invariance principle [15], if *R*_1_ ≤ 1 < *R*_0_, then the equilibrium *E*_1_^*^ is globally asymptotically stable. This completes the proof.

**Theorem 6 .**

Suppose that the conditions (*H*_1_)–(*H*_4_) are satisfied. Then the equilibrium *E*_2_^*^ is globally asymptotically stable if *R*_1_ > 1.

**Proof**

Define a Lyapunov functional

(42) $$\begin{array}{c} U_{2}=W_{3}+W_{4}, \end{array}$$

where

(43) W3=∫T2∗T1−fT2∗,V2∗fσ,V2∗dσ+1k1I2∗gII2∗ +V2∗Nk1k2gVV2∗+qNgk1k2B2∗gBB2∗,

(44) W4=1k1fT2∗,V2∗V2∗∫0h1P1τe−m1τ ×∫t−τtgfTσ,VσVσfT2∗,V2∗V2∗dσdτ +δk1k2I2∗∫0h2P2τe−m2τ∫t−τtgIσI2∗dσdτ,

where *k*_1_ and *k*_2_ are given in (11).

The function *U* : *T* → ∫_*T*_2_^*^_^T^(1 − (*f*(*T*_2_^*^, *V*_2_^*^)/*f*(*σ*, *V*_2_^*^)))*dσ* verifies

(45) $$\begin{array}{c} \dot{U}\left(T\right)=1-\frac{f\left(T_{2}^{*},V_{2}^{*}\right)}{f\left(T,V_{2}^{*}\right)}. \end{array}$$

From (*H*_2_), we have $\dot{U}(T)<0$ for *T* ∈ (0, *T*_2_^*^), $\dot{U}(T)>0$ for *T* ∈ (*T*_2_^*^, *∞*), and $\dot{U}\left(T_{2}^{*}\right)=0$, so *U*(*T*) ≥ 0. Consequently *U*_2_ is nonnegative defined with respect to the endemic equilibrium *E*_2_^*^, which is a global minimum.

We now prove that the time derivative of *U*_1_ is nonpositive. Calculating the time derivative of *W*_1_ along the positive solutions of (2), we obtain

(46) W˙3=1−fT2∗,V2∗fT,V2∗T˙+1k11−I2∗II˙ +1Nk1k21−V2∗VV˙+qNgk1k21−B2∗BB˙=1−fT2∗,V2∗fT,I2∗,V2∗Λ−dT−fT,VV +1k11−I2∗I∫0h1P1τe−m1τfTτ,VτVτdτ−δI +1Nk1k21−V2∗VNδ∫0h2P2τe−m2τIτdτkkkkkkkkkkkkkkkkkkk−cV−qBV∫0h2 +qNgk1k21−B2∗BgBV−μB.

At *E*_2_^*^, by using Λ = *dT*_2_^*^ + *f*(*T*_2_^*^, *V*_2_^*^)*V*_2_^*^, *c* = (*Nδk*_2_ *I*_2_^*^/*V*_2_^*^) − *qB*_2_^*^, and *V*_2_^*^ = *μ*/*g*, we have

(47) W˙3=1−fT2∗,V2∗fT,V2∗dT2∗−dT +fT2∗,V2∗V2∗1−fT2∗,V2∗fT,V2∗−fT,VV +fT2∗,V2∗fT,V2∗fT,VV+1k1∫0h1P1τe−m1τ ×fTτ,VτVτdτ−δk1I+fT2∗,V2∗fT,V2∗fT,VV +1k1∫0h1P1τe−m1τfTτ,VτVτdτ−δk1I −1k1I2∗I∫0h1P1τe−m1τfTτ,VτVτdτ+δk1I2∗ +δk1k2∫0h2P2τe−m2τIτdτ−qNk1k2BV −δk1k2V2∗V∫0h2P2τe−m2τIτdτ+qV2∗Nk1k2B −1Nk1k2V−V2∗Nδk2I2∗V2∗−qB2∗ +qNk2k2B−B2∗V−V2∗=1−fT2∗,V2∗fT,V2∗dT2∗−dT +fT2∗,V2∗V2∗1−fT2∗,V2∗fT,V2∗−fT,VV +fT2∗,V2∗fT,V2∗fT,VV+1k1∫0h1P1τe−m1τ ×fTτ,VτVτdτ−δk1I+fT2∗,V2∗fT,V2∗fT,VV +1k1∫0h1P1τe−m1τfTτ,VτVτdτ−δk1I −1k1I2∗I∫0h1P1τe−m1τfTτ,VτVτdτ+δk1I2∗ +δk1k2∫0h2P2τe−m2τIτdτ−qNk1k2BV −δk1k2V2∗V∫0h2P2τe−m2τIτdτ+qV2∗Nk1k2B −δI2∗k1v2∗V+qB2∗Nk1k2V+δk1I2∗−qV2∗B2∗Nk1k2 +qNk1k2BV−qV2∗Nk1k2B−qB2∗Nk1k2V+qB2∗V2∗Nk1k2=1−fT2∗,V2∗fT,V2∗dT2∗−dT +fT2∗,V2∗V2∗1−fT2∗,V2∗fT,V2∗ −fT,VV+fT2∗,V2∗fT,V2∗fT,VV +1k1∫0h1P1τe−m1τfTτ,VτVτdτ−δk1I −1k1I2∗I∫0h1P1τe−m1τfTτ,VτVτdτ +δk1I2∗+δk1k2∫0h2P2τe−m2τIτdτ −δI2∗k1V2∗V−δk1k2V2∗V∫0h2P2(τ)e−m2τIτdτ+δk1I2∗.

Calculating the time derivative of *W*_4_, we obtain

(48) W˙4=1k1fT2∗,V2∗V2∗∫0h1P1τe−m1τ ×fT,VVfT2∗,V2∗V2∗−fTτ,VτVτfT2∗,V2∗V2∗kkkkkk+ln⁡fTτ,VτVτfT,VVdτ +δk1k2I2∗∫0h2P2τe−m2τII2∗−IτI2∗+ln⁡IτIdτ=fT,VV−1k1∫0h1P1τe−m1τfTτ,VτVτdτ +1k1fT2∗,V2∗V2∗∫0h1P1τe−m1τln⁡fTτ,VτVτfT,VVdτ +δk1I−δk1k2∫0h2P2τe−m2τIτdτ +δk1k2I2∗∫0h2P2(τ)e−m2τln⁡IτIdτ.

Combining (47) and (48) and by using (*δ*/*k*_1_)*I*_2_^*^ = *f*(*T*_2_^*^, *V*_2_^*^)*V*_2_^*^, we obtain

(49) U˙2=1−fT2∗,V2∗fT,V2∗dT2∗−dT +fT2∗,V2∗V2∗1−fT2∗,V2∗fT,V2∗ +fT2∗,V2∗fT,V2∗fT,VV−1k1I2∗I∫0h1P1τe−m1τ ×fTτ,VτVτdτ+fT2∗,V2∗V2∗ −fT2∗,V2∗V−1k2fT2∗,V2∗V2∗I2∗V2∗V ×∫0h2P2τe−m2τIτdτ+fT2∗,V2∗V2∗ +1k1fT2∗,V2∗V2∗∫0h1P1τe−m1τ ×ln⁡fTτ,VτVτfT,VVdτ+1k2fT2∗,V2∗V2∗ ×∫0h2P2τe−m2τln⁡IτIdτ=1−fT2∗,V2∗fT,V2∗dT2∗−dT +fT2∗,V2∗V2∗fT,V2∗fT,V−VV2∗ ×1−fT,VfT,V2∗+fT2∗,V2∗V2∗ ×1−fT2∗,V2∗fT,V2∗+ln⁡fT2∗,V2∗fT,V2∗ +fT2∗,V2∗V2∗1−fT,V2∗fT,V+ln⁡fT,V2∗fT,V +1k1fT2∗,V2∗V2∗∫0h1P1τe−m1τ ×1−fTτ,VτVτI2∗fT2∗,V2∗V2∗I+ln⁡fTτ,VτVτI2∗fT2∗,V2∗V2∗Idτ +1k2fT2∗,V2∗V2∗∫0h2P2τe−m2τ ×1−IτV2∗I2∗V+ln⁡IτV2∗I2∗Vdτ=d1−fT2∗,V2∗fT,V2∗T2∗−T+fT2∗,V2∗V2∗ ×fT,V2∗fT,V−VV2∗1−fT,VfT,V2∗ −fT2∗,V2∗V2∗gfT2∗,V2∗fT,V2∗ −fT2∗,V2∗V2∗gfT,V2∗fT,V −1k1fT2∗,V2∗V2∗∫0h1P1τe−m1τ ×gfTτ,VτVτI2∗fT2∗,V2∗V2∗Idτ −1k2f(T2∗,V2∗)V2∗∫0h2P2(τ)e−m2τgIτV2∗I2∗Vdτ.

From (*H*_2_), we have

(50) $$\begin{array}{c} \left(1-\frac{f\left(T_{2}^{*},V_{2}^{*}\right)}{f\left(T,V_{2}^{*}\right)}\right)\left(T_{2}^{*}-T\right)\leq 0, \end{array}$$

and from (*H*_3_) and (*H*_4_) we have

(51) $$\begin{array}{c} \left(\frac{f\left(T,V_{2}^{*}\right)}{f\left(T,V\right)}-\frac{V}{V_{2}^{*}}\right)\left(1-\frac{f\left(T,V\right)}{f\left(T,V_{2}^{*}\right)}\right)\leq 0, \end{array}$$

and as *g* is positive, we have

(52) $$\begin{array}{c} {\dot{U}}_{2}\leq 0. \end{array}$$

Thus, the equilibrium *E*_2_^*^ is stable. In this case, note that ${\dot{U}}_{2}=0$ if and only if *T* = *T*_2_^*^, *I* = *I*_2_^*^, and *V* = *V*_2_^*^ and using the third equation of (2), we obtain *B* = *B*_2_^*^. Therefore, it follows from LaSalle's invariance principal [15] that the infected equilibrium with *B* cells response *E*_2_^*^ is globally asymptotically stable. This completes the proof.

## 6. Application

In this section, we give some particular examples. In (2), if *f*(*T*, *V*) = (*βT*/(1 + *αV*)) we obtain the following model:

(53) dTtdt=Λ−dTt−βTtVt1+αVt,dItdt=∫0h1P1τe−m1τβTt−τVt−τ1+αVt−τdτ−δIt,dVtdt=Nδ∫0h2P2τe−m2τIt−τdτkkkkkkkk−cVt−qBtVt,dB(t)dt=gB(t)V(t)−μB(t),

The global dynamics of model (53) is studied by Elaiw et al. [5]. So the work presented in [5] is a particular case of (2) because the function (*βT*/(1 + *αV*)) satisfies the hypothesises (*H*_1_)–(*H*_4_).

Another particular case of (2), if *f*(*T*, *V*) = (*βT*/(1 + *aV* + *bT*)) and *h*_1_ = *h*_2_ = *∞*, we obtain the following model which is presented by Yang et al. [13]:

(54) dTtdt=Λ−dTt−βTtVt1+aVt+bTt,dItdt=∫0∞P1τe−m1τβTt−τVt−τ1+aVt−τ+bTt−τdτ   −δIt,dVtdt=Nδ∫0∞P2τe−m2τIt−τdτ−cVtkkkkkkkk−qBtVt,dB(t)dt=gBtVt−μBt.

The global asymptotic stability of possible equilibrium of (54) is established in [13].

A last example, in (2), if *f*(*T*, *V*) = (*βT*/(1 + *αV*)) and *P*_1_(*τ*) = *P*_2_(*τ*) = *δ*(*τ*), where *δ*(·) is the Dirac delta function, we obtain the results presented in [6].

## 7. Conclusion

In the current paper, we have studied an HIV-1 infection model with humoral immune response and intracellular distributed delays and general incidence rate. The model has two distributed time delays describing time needed for infection of cell and virus replication. The global stability of our model is studied by employing the method of Lyapunov functionals which are motivated by McCluskey [16] for delayed epidemic models. This general incidence represents a variety of possible incidence functions that could be used in virus dynamics model as well as epidemic models. We establish that the global dynamics are determined by two threshold parameters, the basic reproduction ratios for viral infection and humoral immune response *R*_0_ and *R*_1_, respectively, which depend on the incidence function and the delay. We have proved that the infection-free equilibrium *E*_0_^*^ is globally asymptotically stable if the basic reproduction ratios viral infection *R*_0_ ≤ 1. In this case, the virus is cleared up. The hypotheses on the general incidence function are used to assure the existence of infected equilibrium without *B* cells response *E*_1_^*^ and infected equilibrium with *B* cells response *E*_2_^*^. We prove that if *R*_1_ ≤ 1 < *R*_0_, the infected equilibrium without *B* cells response *E*_1_^*^ is globally asymptotically stable and if *R*_1_ > 1, the infected equilibrium with *B* cells response *E*_2_^*^ is globally asymptotically stable.
